# Synaptic Plasticity, a Prominent Contributor to the Anxiety in Fragile X Syndrome

**DOI:** 10.1155/2016/9353929

**Published:** 2016-04-28

**Authors:** Tao Yang, Huan Zhao, Changbo Lu, Xiaoyu Li, Yingli Xie, Hao Fu, Hui Xu

**Affiliations:** ^1^Department of Neurobiology and Collaborative Innovation Center for Brain Science, School of Basic Medicine, Fourth Military Medical University, Xi'an 710032, China; ^2^Heze Municipal Hospital, Heze, Shandong 274000, China

## Abstract

Fragile X syndrome (FXS) is an inheritable neuropsychological disease caused by expansion of the CGG trinucleotide repeat affecting the* fmr1* gene on X chromosome, resulting in silence of the* fmr1* gene and failed expression of FMRP. Patients with FXS suffer from cognitive impairment, sensory integration deficits, learning disability, anxiety, autistic traits, and so forth. Specifically, the morbidity of anxiety in FXS individuals remains high from childhood to adulthood. By and large, it is common that the change of brain plasticity plays a key role in the progression of disease. But for now, most studies excessively emphasized the one-sided factor on the change of synaptic plasticity participating in the generation of anxiety during the development of FXS. Here we proposed an integrated concept to acquire better recognition about the details of this process.

## 1. Introduction

Fragile X syndrome (FXS) is the most common mental disorder caused by a CGG trinucleotide amplification on Xq27.3 in the 5′ untranslated region of* fmr1* gene cloned and named in 1991, which suppresses production of fragile X mental retardation protein (FMRP) [1, 2]. FMRP is widely expressed in neuron and glia in brain and acts as an “interactor,” regulating mRNA shuttling, translational control, and synaptic plasticity in copious encephalic regions which are responsible for cognition, emotions, and memory.

In FXS individuals, compared to attention deficits and hyperactivity which were common in childhood but declined remarkably throughout adolescence and adult years, the morbidity of anxiety remains high with impaired ability of information process [3]. It is consistent with the common viewpoint that anxiety is a long-lasting response to danger signals that are either from immediate circumstances or from vague indications of ill-defined events. In short, anxiety is derived from anomalous regulation of fear.

In addition, as one major mood disorder associated with FXS, anxiety occurs with premutation (alleles between 55 and 200 CGG repeats) or full mutation (alleles that exceed 200 CGG repeats) in both genders and affects limbic system and neocortex [4, 5]. Specifically, limbic system and paralimbic system participate in formation and maintenance of anxiety associated with FXS which mainly involve amygdala, prefrontal cortex (PFC), insula, cingulate cortex, temporal cortex, and hippocampus, etc. [6]. Up to now, among all relevant encephalic regions, amygdala–insula is found to be the location where 5-HTTLPR (5-hydroxytryptamine transporter linked polymorphic region) might cause anxiety [7]. The hypofunction of prefrontal cortex and anterior cingulate cortex supports the top-down control mechanisms of anxiety process in affected individuals [8]. The frontostriatal deficits and the dysfunction of the frontoparietal network are proposed to be critical for anxiety processing of external stimuli, etc. [9, 10].

Besides the complicated neural network with abnormal expression of FMRP, the dysgenesis of dendritic spine also significantly influences the synaptic plasticity which accounts for anxiety disorders associated with the development of FXS. And dysfunctional circuits could lead to abnormal spines and vice versa, so it is difficult to figure out which one comes first. Because of intricate involvement of proteins regulated by FMRP in synaptic plasticity through maintenance of spine shape and dynamics, the two defects are arguably inseparable. In the present review, we explored how structure and function coordinately work to promote the anxiety process in FXS and emphasized the selective and monolithic modulation model of the progression.

## 2. Alterations of Synaptic Plasticity in Broad Brain Areas Associated with Anxiety in FXS

Plasticity is considered as a critical process in pain, learning, memory, emotion, cognition, and so on [11, 12]. Substantial evidences have demonstrated that structural changes coordinated with functional changes induce synaptic plasticity, in which LTP and LTD are reciprocally modified by spine density and morphology in* fmr1*-knockout (KO) mice [13–16]. Taken together, change of plasticity induced by defects in spine morphology or neural circuits is significantly involved in the process of anxiety in FXS [16, 17].

On the one hand, it is a significant symbol that the affected individuals have increased quantity of longer dendritic spines. Also, it has been reported that spines were altered in very young* fmr1*-KO mice [18], although spine alterations disappear in adolescent mice [19] and reappear in adult [20, 21]. The inconsistency might be interpreted by postnatal development and regional difference of brain. So far, these observations were acquired in traditional areas, while high-level cognitive regions had not received enough attention. Comparative study in more brain regions of* fmr1*-KO mice is required to fully address this question. FMRP plays a vital role in activity-dependent synapse elimination [22], as well as in spine stabilization [23], to increase the cell-autonomous spine density [18, 24]. For example, in mouse model of FXS, spine density and morphology are altered in an age-, region-, and cell type-specific pattern (Table 1).

On the other hand, it is widely acknowledged that LTP and LTD are molecular mechanisms underlying cognition and emotion. Previous studies showed enhanced metabotropic glutamate receptor- (mGluR-) LTD and impaired cortical LTP in* fmr1*-KO mice. Group I mGluRs are linked to translational activation in neurons and stimulate rapid synthesis of FMRP at synapses. Due to the link of mGluRs with FMRP, mGluR-dependent LTD was enhanced in hippocampus [25–27] and cerebellum [27] in* fmr1*-KO mice. Moreover, cortical LTP is known to be impaired in learning and fear/anxiety memory, including both mGluR-dependent and NMDAR-dependent LTP. And it is expectable that deficits in mGluR-dependent LTP and non-mGluR-dependent LTP in the anterior cingulate cortex and amygdale were correlated with anxiety-like behaviors of FXS [13, 28–30]. Interestingly, the activation of mGluR5 is involved in the late phase LTP (L-LTP) and synaptic depotentiation [29]. This plasticity induced by mGluRs is not simply the alteration of synaptic strength but the change of inducibility of later synaptic plasticity, which suggests that the activation of mGluR5 regulates the transport and function of NMDA receptor [30, 31]. Furthermore, FMRP induced by activation of mGluR5 could be the common molecular mechanism of these phenomena by regulation of transport of NMDA and AMPA receptors [31–33]. Therefore, these results suggest that the lack of FMRP may impair LTP and attenuate cortical network recruitment. Together, the loss of FMRP may participate in cortical LTP deficits via AMPA receptors internalization at postsynaptic neuron.

Taken together, dysgenesis of dendritic spine and deficits of synaptic plasticity result in the formation of anxiety in FXS mouse models. Spine density and morphology have an alteration by an age-, region-, and cell type-specific manner. Also, the defect in spine maturation and pruning is correlated to dysfunction of neural circuits and deficits of synaptic plasticity [16]. On the other hand, deficits of synaptic plasticity as a chronic process contribute to dysgenesis of dendritic spine. Thus, the AMPA receptor internalization, the inheritable rescue of mGluR-LTD, and the rescue of the specific dendritic spine might share the common mechanistic basis. In brief, dendritic spine dysgenesis and defects in synaptic plasticity promote each other in a structure-function interdependent manner.

## 3. Molecular Mechanisms on Synaptic Plasticity Regulated via FMRP

In human genetics, the CGG expansion in the promoter region, which includes the CpG island of* fmr1* gene, is hypermethylated and provokes the silencing of the transcription of the* fmr1* gene, leading to the absence of FMRP, while in the KO mouse model, it is the classical gene knockout effects that result in the silence of fmr1 gene and the loss of FMRP, synaptic function, and plasticity. What is more, recent laboratory studies have provided increasing evidence for the role of FMRP in translational suppression via ribosomal stalling and microRNA [57, 58]. And more evidence about the characteristic of FMRP, a polyribosome-associated RNA-binding protein, reveals more profound mechanisms relevant to abnormal synaptic plasticity. Furthermore, FMRP does not regulate single synapse; instead, it regulates cell-to-cell connectivity. Specifically, at synapses involved in specific situation, two neurons are simultaneously removed, retained, or matured, where FMRP ultimately cause dysfunctional consequences. There are two main theories illustrating the interaction of FMRP and neuronal activity in the cortical circuits.

### 3.1. mGluRs-Dependent or -Independent Synaptic Plasticity Attribute to Anxiety Process in FXS

The anomalous functions of mGluRs-dependent synaptic plasticity have been observed in hippocampus of* fmr1*-KO mice [26, 59, 60]. Activity-dependent synthesis of FMRP in enduring forms of synaptic plasticity may be induced via exaggerated mGluR-LTD in hippocampal neurons, while the initiation of long-term potentiation (LTP) is a qualitatively different functional consequence of Group I mGluR-stimulated protein synthesis at the synapses of hippocampus where LTD can be induced [25, 29]. Besides, the mGluR theory proposes that stimulation of Group I mGluR induces local mRNA translation, resulting in novel protein synthesis that subsequently enhances the internalization of AMPA receptors [61, 62]. This model predicts that, in absence of FMRP, the increased translation of a subset of mRNAs disturbs receptor internalization dynamics and then exaggerates internalization of AMPA receptors and weakens the synapse. What is more, independent protein synthesis mGluR-LTD in* fmr1*-KO mice suggests that in absence of FMRP, proteins that are significant for the maintenance of mGluR-LTD are already largely present at the synapses. Overall, the mGluR theory presents a well-defined mechanism of anxiety in FXS by all accounts: higher density of spines and more immature spines which lead to deficits and anxiety-like behavioral phenotypes in FXS. The mGluR-LTD theory was considered as the main theory of psychological symptoms associated with FXS [26, 61]. Moreover, the mGluR theory has directed research towards the preclinical mechanisms underlying FXS and led to the effective novel therapeutic strategies [31, 63–66].

From the further intracellular perspective, the phosphorylation of FMRP influences the translation of target mRNAs because unphosphorylated FMRP is associated with actively translating polyribosomes while phosphorylated FMRP is associated with inactive polyribosomes [67]. By and large, there are three signaling pathways downstream of mGluR5 affecting translation: the PI3K-mTOR, the MEK-ERK-Mnk1, and the CaMKIV-CREB pathways. Activation of mammalian mTOR cascade results in the phosphorylation of protein phosphatase 2A (PP2A) and S6 kinase [68] and mRNA translation rapidly [60]. Besides, a thesis reported enhanced Ras-PI3K signaling input induced by the activation of GluA1 enriches the mTOR signaling pathway [52]. Thus, the overactivated mTOR signaling pathway in the hippocampus might play a prominent role in FXS. However, no analogy is reported to compare the relationship between NMDA and mTOR signaling. More efforts are required to supply the signaling and to explore more potential targets. Also, it has been demonstrated that cAMP responsive element-binding protein (CREB) contributed to the regulation of FMRP by Group I mGluRs and was closely linked to anxiety [55, 69]. Therefore, the main three signaling pathways work together downstream of mGluR5 to influence the protein synthesis, synaptic plasticity, and anxiety-like behaviors (Figure 1).

What is more, the cAMP theory was proposed as a supplement to mGluR theory [70]. Apparently it is a potential shortcoming in the context of the mGluR theory; Ca^2+^ and PKC are both part of the Gq cascade, which are able to regulate certain AC isozymes and disrupt normal function. Also, there are evidences that cyclic AMP and mGluR interact with each other because G protein has the potential to act through a network of multiple overlapping messengers [71]. Furthermore, the fact that mGluR inhibitors rescue cAMP deficits in FXS and presumably downstream of excessive mGluR activity [72] supports the idea that the two theories operate in series.

### 3.2. Dysfunctional GABAergic Synaptic Plasticity in Interneurons Modulates the Pathological Anxiety in FXS

Another significant pathway was GABAergic neurons. Importantly, FMRP is broadly expressed in GABAergic neurons [73], indicating that it is involved in normal interneuron maturation and function modulation. Indeed, it is significant that GABA can modulate neurotransmitter release in an autocrine or paracrine fashion, via mechanisms at presynaptic GABA_A_ and GABA_B_ receptors [74, 75]. For example, on the presynaptic side, where FMRP is also expressed [76, 77], the expression of GABA-synthesizing enzyme GAD in* fmr1*-KO mice is found increased or decreased [73, 78–81], with the change relying on the brain region examined.

In summary, GABAergic signaling is essential for regulating neuronal migration, maturation, and circuit formation. And defects in the GABAergic system are, therefore, likely to have profound effects on neuronal development and circuit function in FXS. Currently, a better understanding of early developmental alterations in GABAergic system in FXS would be reckoned as the crucial insight into the nature of the FXS brain, as well as valuable information about key pharmacological targets. Furthermore, in mature neurons, the ionotropic GABA_A_ receptors mediate postsynaptic hyperpolarization via intracellular Cl^−^ influx, while GABA_B_ receptors activation likewise hyperpolarizes the postsynaptic membrane by activating G-protein-coupled inwardly rectifying K^+^ channels. In addition to its role as a postsynaptic inhibitory neurotransmitter, distinct mechanisms modulate neurotransmitter release at presynaptic GABA_A_ and GABA_B_ receptors [74, 75]. Meanwhile, over behavioral effects, GABA_A_ receptors seem to affect more short-term plasticity, seizures, learning and memory deficits, and poor motor skills on a repetitive task and hyperactivity features [42, 82, 83]. And GABA_B_ receptors more likely result in social impairment. For instance, papers have reported STX209, a GABA_B_ agonist, might improve neurobehavioral function and satisfying effects were obtained in a phase 2 trial [42, 82]. It also worth noting that the role of GABA in the developing CNS is dynamic and variable between brain regions. Therefore, the same GABAergic effectors that helped adult patients could have adverse effects in developing individuals based on the function of GABA in particular brain regions at specific developmental time periods.

### 3.3. Probable Relationship between Abnormal mGluRs and GABA Synaptic Plasticity

Overall, both abnormal mGluRs and GABA synaptic plasticity play significant synergistic roles in the formation of anxiety. The GABA_B_ receptor may serve as the functional link between both pathways, as this metabotropic receptor regulates glutamate release at glutamatergic synapses. In FXS patients, a reduced release of GABA from the GABAergic terminals to the presynaptic GABA_B_ receptors may induce a reduced inhibition of neurotransmitter spillover, which in turn activates mGluR signaling [84]. One mechanism of modulating GABA release involves the synthesis and mobilization of endocannabinoids [85]. Activation of Group I mGluRs enables mobilization of endocannabinoids in the postsynaptic neuron and negatively modulates GABA release through a mechanism known as depolarization-induced suppression of inhibition (DSI) [86, 87] (Figure 2). These mechanisms require increased neuronal activity, which exists in brain circuitry of* fmr1*-KO mice [88]. Therefore, in consideration of endocannabinoid mobilization in the FXS, the loss of FMRP may selectively affect specific inhibitory circuits. In the developing and mature brain, it is critical for cortical excitatory neurons to be proper synchronized at behaviorally relevant frequencies [89–92]. And thus, alteration of mGluR signaling in this specific type of interneuron is likely to have wide-reaching effects in developing and mature cortical networks and needs to be further explored.

## 4. Possible Definitions of Diverse Functional Synaptic Plasticity Phenotypes between Hippocampus and Other Regions

How LTP deficits and enhanced LTD are temporally and spatially coordinated with each other in different regions remains to be determined. From the intrinsic modulation perspective, it has been showed that FMRP would suppress the translation stimulated by neuronal activity and generate neuronal feedback responses to activity at the neuron level. Adding to suppression of translation by miRNA and stalled polyribosomes, synaptic regulation, which involves glutamate receptor signaling, GABA receptor signaling in neurons, and intracellular PKA, PKC, cAMP, and PI3K signaling pathways, also implicates FMRP. But this cannot define the complicated plasticity well. Here we would like to illustrate this problem involving receptors and cascade signaling sides.

On the one hand, mGluR and NMDA subtypes, as FMRP targets, have diverging structure and features, determining diverse downstream signaling targets, as described before. Besides, the initial “interactor” role of FMRP associated with its transcripts targets needs more attention. From stimulated receptors on neurons to intracellular signaling, it could be conclusive that FMRP selectively regulates the expression of components of the ERK and mTOR signal transduction pathways in different brain areas. For example, activating GluA1 results in the downstream Ras-PI3K signaling in hippocampus which shares Ras protein with mTOR signaling [52]. And these signalings convert receptor activity into translational output. Taken together, it seems that FMRP associated with its target transcripts directly regulates translational control of the pre- and postsynaptic proteome and synaptic plasticity in different brain areas.

Considering the primary and secondary procedures, the process should be examined at different times of the nucleus modulation, mRNA, or proteome life-cycle. Previously, it has been proposed that RNA interference and stalled polyribosomes implicate FMRP. As for now, miRNA family, including miR-125b, miR-132 [93], and miR-196a [94], were found to be relevant to the regulation. Furthermore, using Moloney leukemia virus (MOV10) to unfold the structured Argonaute 2 (AGO2) through RNAi [95] and adenosine-to-inosine RNA-editing [96, 97] proposed novel perspectives to explore the widely unknown target RNAs and associated regulation pathways. Meanwhile, recently, a sensational work reported that Cdh1-anaphase-promoting complex (APC) and Cdc20-anaphase-promoting complex control the morphogenesis of axons and dendrites and synaptic plasticity. Cdh1-APC and FMRP are components of a novel ubiquitin signaling pathway that regulates mGluR-LTD in brain in terms of cell cleavage or neuronal development [98]. Together, an original work reported that the* Drosophila* fragile X homolog (dFMR1) biochemically interacted with the adenosine-to-inosine RNA-editing enzyme dADAR [96, 97]. And all this work may propose an original view of nucleus modulation of FMRP and consummate the cognition of FMRP's interactor role on DNA, mRNA, and stalled polyribosomes levels. Therefore, we can conclude that the cleavage and differentiation of neuron, involving gene editing, RNAi, and stalled polyribosomes are integrated and implicated patterns. And just these manners interfere with the diverse synaptic plasticity between hippocampus and other regions.

## 5. Future Prospects in Defining the Complicated Neuropsychological Behaviors and the Mechanisms of Anxiety in FXS

Generally, anxiety is caused not only by connate factors but also by self-regulation of brain homeostasis. During propofol sedation, FXS subjects have significantly decreased the rates of cerebral protein synthesis (rCPS) in brain as a whole, cerebellum, and parts of cortex, which also suggests changes in synaptic signaling can balance increased rates of cerebral protein synthesis (rCPS) in FXS [57]. Also, considerable laboratory research has accumulated copious evidences based on the changes of synaptic plasticity associated with anxiety. However, there also exist contradictory and promising fields to explore:

1. While further data linking these morphological changes to the functional modifications underlying anxiety process were relatively lacking in FXS, a potential entry point to it is the BDNF-TrkB signaling [15]. Also, given the respective importance of AMPARs and the Rho GTPases in functional and morphological plasticity [99], the exploration of interactions between these two signaling pathways may provide a mechanism to illustrate these changes.
2. Short-term plasticity (STP) is widely believed to play a key role in synaptic information transmission by optimizing the neural output in response to specific patterns of neuronal activity [100]. Although it was identified that presynaptic actions in hippocampus are mediated by the large conductance Ca^2+^ activated K^+^ (BK) channel together with the interaction of FMRP [53], further study is needed.
3. In recent years, the development of iPSCs (induced pluripotent stem cells) technology is emerging flourishingly. A typical example is that generation of naive/ground state FXS-iPS cells with reactivated FMR1 successfully figure out a mechanism of transcriptional silencing. In this mechanism, FMRP might direct binding the RNA-induced silencing complex (RISC) on the FMR1 transcript and lead to production of 22–26 nt CGG fragments. And then it facilitates FMR1 methylation and silencing by directing histone modifying proteins to the locus [101].
4. Proteins play a complicated role in organisms extensively. Lately, a sensational study published in* Science* firstly reported that Rqc2 can promote alanine and threonine synthesizing uncompleted protein without the manipulation of DNA and mRNA [102]. Meanwhile, this peculiar phenomenon may also occur in FXS because of its specific stalled polyribosomes. Or maybe some special proteins having homogeneous functions remain to be explored.

## 6. Summary

Synaptic plasticity reveals flexibility and codes capacity of neuronal networks. In FXS, the absence of FMRP perturbs the balance in array of diverse plastic mechanisms of synaptic plasticity in a developmental and regional dependent way. And along anxiety process, a very close structure-function relationship exists between spines and neuronal activity: synaptic strength, synaptic forms of plasticity involved in learning and memory, and activity-dependent plasticity. From the morphology and structural perspectives, increased density of longer immature spines may induce the synaptic plasticity and may result from the loss of FMRP in multiple interlaced brain areas. On the point of molecular mechanisms underlying alterations of synaptic plasticity, the proteins encoded by FMRP target mRNAs indicate a high level of control over the balance of activity-dependent translation in synaptic plasticity. First, mGluR and NMDAR-dependent synaptic plasticity are altered in FXS mouse models [45, 62]. Specifically, this dysregulation of processes involves downstream of Gp I mGluR signaling and AMPA receptor internalization, GABA release, and regulation of mGluRs and GABA via endocannabinoid. Second, FMRP regulates the expression of components of the ERK and mTOR signal transduction pathways selectively, but not in only one way (Table 2).

Finally, gene editing, endogenous RNAi, and stalled polyribosomes may influence the internal regulation of synaptic plasticity. Or just this integrated regulation, not single targets, facilitates the pathological progression of plasticity and anxiety-like behavior in FXS.

## Figures and Tables

**Figure 1:** Signaling pathways downstream of Group I mGluR stimulation. There are three signaling pathways downstream of mGluR5 affecting translation: the typical PLC cascade reaction, the MEK-ERK-Mnk1, and the PI3K-mTOR pathway. Activation of mTOR is one of the primary triggers for the initiation translation via phosphorylation of 4E-BP and S6K. After stimulation of mGluR5, PI3K phosphorylates the membrane phospholipid PIP2, converting it to PIP3. PIP3 recruits Akt to the membrane and then Akt activates mTOR by inhibiting TSC. Subsequently, mTOR interacts with Raptor, which binds both 4E-BP and S6K. Phosphorylation of S6 and 4E-BP finally results in mRNA translation. ERK is a point of convergence of several signaling cascades. Several FMRP target mRNAs (PP2A and PI3K) are members of second messenger cascades converging on ERK. ERK phosphorylation is regulated by phosphatases such as PP2A. In* fmr1*-KO mice, PP2A is overactivated after mGluR5 stimulation, causing the rapid deactivation of ERK. The Ca^2+^ stored by IP3 release leads to activation of Ca^2+^-calmodulin (CaM) dependent pathways, including AC1-cAMP dependent protein kinase (PKA) and CaMKIV, which were stimulated by CaM and then phosphorylate CREB. Phosphorylated CREB initiates the CREB-dependent transcription of* fmr1* gene and upregulates FMRP. MEK, mitogen-activated protein kinase kinase; ERK, extracellular signal regulated kinase; Mnk1, mitogen-activated protein kinase interacting serine/threonine kinase 1; PI3K, phosphoinositide-3 kinase; 4E-BP, 4E-binding protein; S6K, S6 kinase; PIP2, phosphatidylinositol 4,5-bisphosphate; PIP3, phosphatidylinositol (3,4,5)-trisphosphate; TSC, tuberous sclerosis complex; GAP, GTPase-activating protein.

**Figure 2:** Potential patterns linking mGluRs theory and GABA theory which influence synaptic plasticity involving proteins regulated by FMRP. Activation of Gp1 mGluRs enables the mobilization of endocannabinoids (eCB) in the postsynaptic neuron and retrogradely modulates GABA release through a mechanism known as depolarization-induced suppression of inhibition (DSI). In the whole process, Ca^2+^ influx into postsynaptic neuron participates in the mobilization of endocannabinoids, whereas at presynaptic neuron, Ca^2+^ influx into the cytoplasm restrained by endocannabinoids participates in the inhibition of GABA release.

**Table 1:** Spine phenotypes in broad encephalic regions and at different periods. In the mouse model of FXS, spine density and morphology were altered in an age-, region-, and cell type-specific manner.

Brain areas		Methods	Spine phenotypes	Reference
Hippocampus	Development	P0 + 7 DIV or 21 DIV; fixed, Dil	Decreased density Normal length	[34]
		P0 + 16 DIV; fixed, FITC-phalloidin	High density Longer spines More immature and lacked synapse in puncta	[35]
		CA1 and CA3 E15/16 + 14 DIV or P7 Fixed and in vitro, GFP	Density not reported Longer spines at P7 More immature	[36]
		P6/7 + 4-5 DIV Fixed, cultured slices, two-photon, GFP	Normal density Length not reported	[37]
		CA1; 2-week-old; confocal imaging, fixed, Dil	Normal density Decreased spine length	[38]
	Adult	Dentate gyrus granule cells; juvenile-adult (P15–P60); fixed, Golgi, EM	Higher density Length NA More immature	[39]
		CA1; 3-month-old; fixed, Golgi	Higher density Length NA More immature	[40]
		CA1; 10/25-week-old; confocal imaging fixed, Dil	Normal density Longer spines	[38]

Amygdala	Adult	Basolateral amygdala; 3-month-old; fixed, Golgi	Higher density Longer spine More immature	[24, 40]

Cortex layer 2/3	Development	Barrel cortex; P7–P21; in vivo, two-photon, GFP	Normal density Normal length High turnover at P10–12 More immature spines	[23]
		Primary visual cortex; two-week-old; Golgi, fixed	Normal density Longer spines	[41]
		Prefrontal cortex; two-week-old; acute slice, two-photon	Normal density Longer spines	[13]
	Adult	Visual cortex; P35 (±1); Golgi, fixed	Higher density Length NA	[42]
		Temporal cortex Adult (two months) Golgi, fixed	Higher density Normal length (trend toward longer spines)	[43]
		Medial prefrontal cortex; adult (13 weeks); fixed, Golgi	Higher density Longer spines	[44]

Cortex layer 4	Development	Barrel cortex P7, P14; Golgi, fixed	Normal density	[45]

Cortex layer 5	Development	Barrel cortex P7–P21; fixed, two-photon, GFP	Normal density at P14 and P30; high density at P7 Longer at P7 and P14, then normal at P30	[19]
		Barrel cortex P2 + 5 DIV; cultured slices, two-photon, GFP	Normal density Normal length Normal motility	[19]
	Adult	Visual cortex Adult Golgi, fixed	Higher density More immature	[46–48]
		Visual cortex Adult Golgi, fixed	Normal density Length NA More immature	[14]
		Barrel cortex Juvenile and adult Golgi, fixed	Normal density in juvenile (P25); higher in adults Normal length in juvenile; longer in adults More immature	[20]
		Occipital cortex Adult (60–90 days) Golgi, fixed	Higher density Longer spine More immature	[47]

Major drawbacks in comparing these different studies are caused not only by the use of different staining, quantification methods of spines, choice of tissue source, and hippocampal neurons cultured in in vivo or ex vivo brain tissue, but also by different mouse strains. Also, the classification of dendritic protrusions into different categories, such as mature and immature, differs between studies (some look at the presence versus absence of a head, other at the ratio between the width and the length of the protrusion, and also others, at the profile).

BDA, biotinylated dextran; DIV, days in vitro; EM, electron microscopy.

FITC, fluorescein isothiocyanate; Dil, diOlistic labelling.

GFP, green fluorescent protein; NA, not available.

**Table 2:** FMRP selectively regulates signaling pathways associated with transcript targets in different brain regions.

Brain areas	Synaptic plasticity phenotypes	Signaling pathways
Hippocampus	mGluR-LTD	ERK1,2 [49]; mTOR phosphorylation [49]; CB1 signaling [50]
	LTP deficits	PKC-CaMKII [51]; Ras-PI3K/PKB [52]
	Increased STP	Decreased presynaptic BKCa^2+^ channels activity [53]

Amygdala	LTP deficits	cAMP-CREB [28, 54]

ACC	Decreased LTP	CaMKIV [55]

PFC	Impaired LTP	G*α*s-cAMP [56]
